# Evaluation of Posturometric Parameters in Children and Youth Who Practice Karate: Prospective Cross-Sectional Study

**DOI:** 10.1155/2022/5432743

**Published:** 2022-06-26

**Authors:** Anna Brzęk, Andrzej Knapik, Bogusław Brzęk, Paweł Niemiec, Piotr Przygodzki, Ryszard Plinta, Karol Szyluk

**Affiliations:** ^1^Faculty of Health Sciences in Katowice, Department of Physiotherapy Chair of Physiotherapy, Medical University of Silesia in Katowice, 12 Medyków St., 40-752 Katowice, Poland; ^2^Faculty of Health Sciences in Katowice, Department of Adapted Physical Activity and Sport, Medical University of Silesia in Katowice, 12 Medyków St., 40-752 Katowice, Poland; ^3^All4Health Bogusław Brzęk, Dynamic Medical Center, 38 Rakietowa St., 54-615 Wrocław, Poland; ^4^Department of Biochemistry and Medical Genetics, School of Health Sciences in Katowice, Medical University of Silesia in Katowice, Medyków 18 Str., 40-752 Katowice, Poland; ^5^Department of Health Policy, Abbott Laboratories, 21B Postępu Street, 02-676 Warszawa, Poland

## Abstract

Reduced physical activity or inappropriate training can cause the development of postural abnormalities. The aim of the present study was to determine the relationship between intensive, controlled physical activity, such as karate, and postural parameters. The study group consisted of 57 young karate competitors aged 9–12 years. The control group included 76 healthy, active children in similar age. The children's posture, activity level, and time in front of electronic devices were evaluated. The following body posture assessments were carried out: Adams' test, evaluation of the plumb line, evaluation of the kyphosis, and lordosis angles using a digital inclinometer and shoulder blade position measurements using a pediscoliometer. In the majority of cases, despite evidence of an increase or decrease in the values of the plumb line and scapulae level, the results were still within the normal ranges. In 71.93% of the examined karate-training children, a decrease in torso rotation was noted. The study revealed a visible difference in postural muscle strength by the Mathiass screening test (*P* < 0.00001). The children in the control group spent more time in front electronic devices than the karate-training children did (*P* < 0.007). Postural defects regression was more often observed in the study group than in the controls (*P* < 10^−8^). The frequency of postural defects stabilization was also significantly higher in the study group than in the control children (*P* = 0.001). Conversely, postural defects progression was significantly more frequent in the control group than in young karate competitors (*P* < 10^−8^). These differences remained significant in subgroups of girls and boys. Physical activity performed regularly and under the direction of a professional trainer can prevent postural disorders.

## 1. Introduction

Technology development in modern civilization causes lifestyle changes in societies. This includes young people [1]. In addition to many positive changes, some negative changes—from the health point of view—also occur. One of the most important negative changes is a reduction in the level of physical activity (PA), which often decreases to a level below the daily recommendation for good health (MVPA) [2].

Usually, the decrease in PA level is a consequence of children and young people spending increasingly more time in front of a TV, computer, or tablet [3, 4]. WHO recommendation has shown that the optimal level of PA is an essential factor in the proper development of children [2]. Therefore, PA conditions, courses, and consequences are being examined [5, 6]. The definition of the proper body posture points to individual variability, although it is possible to point to some common features defined according to Nowotny by the reciprocal configuration of its particular segments [7]. In the period of posturogenesis, it undergoes characteristic changes with varying degrees of intensity and changes of a more or less dynamic character. Its critical periods of posturogenesis are worth pointing out, during which errors in body posture, generated by rapid growth or, later on, by the development of sexual signs, occur much more frequently. The first critical moment occurs at the age of 6-7 years and the next at puberty (11-14 years depending on sex) [7]. Endogenous and exogenous factors influence the quality of posture. During the school stage, the reasons for unfavourable changes in body posture are most often attributed to new, previously unknown school conditions and factors, such as unfavourable static postures (e.g., staying in desks for many hours) and unfavourable physical and mental conditions school, carrying additional loads (school bags filled with heavy books) [8], psychological factors (e.g. stress), and hygienic-health factors (inactive lifestyle) [9]. The pubertal leap period, on the other hand, was identified as critical due to the high developmental disharmony occurring at this time [8].

The negative consequences of a lack of a sufficient level of PA involve biological, functional (motor), psychological, and social aspects. The most frequently mentioned consequences include overweight and obesity [10, 11]; abnormalities in body posture, including serious deformities of the spine [12]; a loss of coordination; poor motor skills; and consequences associated with isolation among peers [13, 14]. Low levels of PA in children and adolescents may be the reason for their reluctance to exercise, which often persists throughout their lives [14].

Among the numerous forms of activities that are offered, martial arts (MA), which are popular worldwide, plays an important role in PA. The importance of practicing MA spans beyond the promotion of physical health. Practicing MA is of great importance for improving psychological well-being [15]. The potential to use MA for the development of various forms of intelligence or as a form of therapy is being studied [16, 17].

One of the sports classified as MA is karate. It has many advantages, so it is recommended for children. The primary advantage of karate is the safety of the exercises [18]. Particular importance is given to the motor development of children practicing karate [19, 20]. Another benefit of practicing karate is lower level of aggression that occurs in children practicing this sport in comparison with their inactive peers or those who practice other sports [21, 22]. Because of the benefits exhibited in children from practicing karate, from the preventive care point of view, it may be interesting to investigate the relationships between this sport discipline and individuals' posture quality.

This problem has been identified but has not been solved yet. Therefore, in this study, the researchers analyzed the benefits of practicing karate among children. The research is only a part of a large scientific project conducted by the first author. The objective for this study was particularly important for children because the behaviors they develop during childhood will become habitual in the future and will play an important role in their quality of life during adulthood.

The aim of the study was to evaluate children's physical activity and body posture. The most important matter was to determine whether there is relationship between intensive, controlled physical activity, such as karate, and posturometric parameters.

Our research will clarify how does a child's body posture change after 11 months of karate training and what is the cause of the above-mentioned changes. We wish to establish how significant it is to implement martial arts for the prophylaxis of body posture disorders. Lastly, we want to answer does regular physical activity influences habits in free time?

## 2. Materials and Methods

### 2.1. Study Design

This prospective observational cross-sectional study was designed in accordance with STROBE guidelines. A cohort of 1,596 children was examined to identify cases characterized by regular physical activity (Figure 1). A number of 207 subjects were qualified for the study and assigned to two groups, namely, the study group, which were young karate competitors who performed karate training 2–3 times a week, and the control group, which were children performed physical activity 2–3 times a week for at least 60 minutes. Posturometric parameters were examined in all children twice, at the beginning of the examination (initial examination) and after 11 months (final examination). The frequency of postural defect regression, stabilization, and progression was then calculated and compared between groups. An assessment of the time spent by children in a sitting position and with electronic devices was also performed. Finally, both stages of the study were completed by 57 children from the study group and 76 children from the control group (Figure 1). Detailed data on the subjects, the inclusion criteria, and the methods used are presented below.

The study was approved by the Ethics Committee of the Medical University of Silesia in Katowice, Poland, under resolution no. KNW/0022/KB1/162/10 and no. KNW/0022/KB1/100/16. It is conformed to the Helsinki Declaration. All patients and their parents/guardians provided written informed consent prior to the study, including enrollment and data collection.

### 2.2. Subjects

The study involved 133 children aged 9–12 years old (mean ± SD: 10.7 ± 1.07). In this group, there were 63 girls and 68 boys from the region of Upper Silesia (Poland). The study group consisted of 57 young karate competitors who performed karate training 2–3 times a week (mean ± SD: 2.63 ± 0.48). They were trained between 60 and 90 minutes per one session (mean ± SD: 76.84 ± 17.94). Among the karate athletes surveyed, there were no children with a dan master's degree. Most were children with the rank of 10-8 kyū, granted for children under 14 yr. Competitors did not practice another sport regularly, other than actively spending free time with their parents. The control group included 76 healthy children, age and sex matched (*P* > 0.05), who declared that they performed physical activity. The trainings were preventive but were not conducted by professional trainers. However, the parents of the children declared the required limit of unit training at least 60 minutes 2–3 times a week (mean ± SD: 66.71 ± 13.54). They spent their active free time performing activities (e.g., swimming, bicycle, skiing, walking, and playing football) with their parents and without a trainer. The children in both groups regularly participated in PE (Physical Education) lessons.

The study was planned on the age group 9-12 years qualified to the younger school age, in which the slowest level of growth is assumed. The group included prepubertal girls and boys with a maximum growth typical for this period of 5-6 cm/year [23, 24]. Girls were not menstruating in both studies. The exclusion criteria involved the diagnosis of scoliosis or other serious posture abnormalities that were present in any of the three planes. These excluded children were referred to an orthopedic specialist for further evaluation. The other exclusion criteria were as follows: age below 9 or above 12, irregular participation in children training sessions, exemption from physical education classes because of frequent infections, orthopedic injuries, or pulmonary diseases (e.g., asthma and allergies). Children who exhibited “growth spurt” (an increase in body height of 7 cm or more between studies), appearance of the first menstrual period, or obesity states that could influence the results of the posture evaluation were also excluded from the study. In the control group, children who had been systematically training a sport discipline other than karate for more than 1 year were excluded from the control group. The number of examined karate children totaled 104, but 57 children were chosen for the final analysis. The remaining participants were excluded from the analysis because of growth spurts, a long absence in karate training and diagnoses of orthopedic injuries during the school year (Figure 1).

### 2.3. Examination

All of the children who qualified for the study were examined in the same conditions by the one experienced and qualified researcher (physiotherapist with ten years of experience as an operator of the equipment and 15 years of experience in testing body posture), who used classic tools and tests used in body posture evaluations [25]. Examination was carried out at two times: first, at the beginning of the school year, after summer (initial examination), and second, after 11 months (final examination). From a detailed examination to further detailed analysis, the following factors were taken into account: body height, body weight, torso rotation angle, kyphosis and lordosis angles, position of the shoulder blades, deflection of the plumb line from the gluteal cleft, and Hump Sum indicator. An analysis of the differences between the following examinations was performed with particular attention to details. The data were analyzed independently for both initial and final examination, and then, these results were compared and evaluated. The BMI values were calculated on the basis of height and weight of the participants and expressed as BMI-for-age percentiles [26, 27].

### 2.4. Posturometric Analyses

Body posture measurements were performed according to the methodology presented below. For the body posture evaluations, the authors used classic tools and tests that have been suggested for use by SOSORT (Society of Scoliosis Orthopaedic and Rehabilitation Treatment), which required a scoliometer, digital inclinometer, or plurimeter plumb line (with certificate). The test-retest reliability *R* value was above 0.846 for each test used. The intraobserver reliability was assessed by Cochran's *Q* test, which yielded *P* > 0.13 for all the tests used. The torso rotation angle was measured in the standing position with a pediscoliometer during the Adams' test (measured three times). The torso rotation angle was measured at three levels: at the cervical kyphosis peak, the thoracolumbar junction, and the lumbar lordosis peak. The highest values of the torso rotation angle from all of the analyzed levels were taken for the study. Based on the obtained results, the Hump Sum indicator was calculated to avoid a mistaken overdiagnosis of body posture abnormalities [28]. Subsequently, the amount of plumb line deflection from the gluteal cleft was evaluated. The plumb line was projected from the external occipital protuberance to the gluteal cleft, and the amount of deflection to the right or left was measured in centimeters. Afterwards, the kyphosis and lordosis angles were measured according to the methodology reported by Brzęk et al. [29] with the use of a digital inclinometer SAUNDERS TMX-127 (Baseline Digital Inclinometer, Saunders Group Inc., Chaska, MN, USA). The pelvis and shoulder blade positions were measured using a ruler and pediscoliometer (by Pedihealth Oy, Finland). The Mathiass test for postural muscle endurance was administered in the standing position with the arms bent to 90° for 30 seconds (Figure 2).

The comparison of the results of posturometric parameters between the initial and final examination was used to assess the regression (decrease of the parameters defined as postural defects), stabilization (no significant changes in body posture parameters between initial and final examination), and progression (increase of the parameters defined as postural defects) of postural defects in both studied groups. The differences in the frequency of each of them were then compared between groups.

### 2.5. Assessment of the Time Spent with Electronic Devices

Each group answered questions regarding how much time they spend with electronic devices. The questions in the author's questionnaire addressed the eventual use of mobile, tablet, PC, and computer games at home or school, during weekdays and weekends. The reported individual time (in minutes) referred to the amount of time that participants spent with each electronic device, separately, and in total. Due to young age and sometimes lack of ability to determine the length of the time period, screen time was assessed by children parents.

### 2.6. Statistical Analysis

Statistica 12.0 software (TIBCO Software Inc., CA, USA) was used for most of the statistical analyzes. All quantitative data were given as a mean, their spread as a standard deviation (SD), and their range. The normality of distribution was checked by the Kolmogorov-Smirnov test. The differences between groups were estimated by a linear regression, which was adjusted for age (most of the analyzed parameters are directly age-related), with a 95% confidence interval (CI). The following statistical methods were used: the Mann–Whitney *U* test for continuous variables with nonnormal distribution, Student's *t*-test for continuous variables with normal distribution, and *χ*^2^ and Spearman's rank tests for nonparametric characteristics. Spearman's rank correlation coefficient (*r*_*s*_) was used as a nonparametric measure of correlation. Fisher's correction was used in comparisons, when the number of subjects was less than ten. The differences of quantitative data of matched samples between the initial and the final examination were computed using the Wilcoxon signed-rank test (for variables with nonnormal distribution) or the Student's *t*-test (for variables with normal distribution). The sample size and the power analysis were computed using the Epi-InfoTM 7.2.1.0 software (Centers for Disease Control and Prevention, USA). The results of statistical tests were considered significant at the level of *P* < 0.05. In the case of multiple comparisons, the Bonferroni correction was applied. Cases with missing data were rejected from the respective comparisons.

## 3. Results

### 3.1. The Overall Characteristics of the Examined Groups

The groups were homogenous, and no statistically significant differences between the groups of girls and boys were noted in terms of their age, height, or weight. The participants' body height ranged from 128 to 171 cm (mean ± SD: 148.22 ± 10.28) in the study group and from 122 to 168 cm (mean ± SD: 146.47 ± 10.77) in the control group (*t* = 0.94; *P* > 0.05). The children' weights ranged from 21.5 to 55.0 kg (mean ± SD: 36.98 ± 7.02) in the study group and between 22 and 55 kg (mean ± SD: 35.59 ± 7.25) in the control group (*t* = 1.10; *P* > 0.05). In the examined groups, the BMI-for-age percentiles ranged between the 3rd and 85th (mean ± SD: 31.26 ± 22.96 in the study group; mean ± SD: 38.98.27 ± 20.77 in the control group).

### 3.2. Body Posture Characteristics in the Initial and Final Examination

The changes in posturometric parameters between the first (initial) and the second (final) examination were noted. The changes concerned all of the examined posturometric parameters in both examined groups (Tables 1 and 2).

In the study group, changes in the obtained results were expected. In the majority of cases, despite an increase or decrease in the values of the plumb line and scapulae level, the results were still within the normal ranges. In 71.93% of the examined karate-training children, a decrease in torso rotation was noted. The sex of the participants did not play a significant role (*χ*^2^ = 5.76, *P* = 0.05, for df = 2). The ATR (angle trunk rotation) changes were not dependent on training frequency (in both groups, Spearman's *r*_*s*_ = 0.01) and training times (-0.18 for the study group and 0.05 for the control group). The Hump Sum indicator depended on the training years only in the control group (Spearman's *r*_*s*_ = 0.25). An increased ATR value was evident in 22.8% of the examined children in the study group and 65.79% of the children in the control group; in 27.63% of examinees, the ATR value was more than 7, and in 19.84%, there was significant asymmetry in the plumb line, scapulae level, and pelvic obliquity, which were not evident in the initial examination. In the present study, the boys obtained much worse results than the girls (*χ*^2^ = 18.49, *P* < 0.02). The children for whom scoliosis was suspected were referred to orthopedic specialists, and further treatment and rehabilitation were recommended. In the study group, in 8 examined children (14.03%), the Hump Sum indicator ranged between 4 and 6 degrees, and these children underwent another assessment within 6 months. Only 5 children (8.77%) in the study group were referred for an orthopedic consultation. The normal ranges of thoracic kyphosis and lumbar lordosis angles, presented by Brzęk et al. [29], were both 24–36 degrees. In total, the criteria were met by 100% of children from the study group and 76.32% of children from the control group.

The frequency of postural defects regression, stabilization, and progression at the final examination are presented in Table 3. Postural defect regression was more often observed in the study group than in the controls (47.36% vs. 4.11%, respectively) and this difference had strong statistical significance (*P* < 10^−8^, *χ*^2^ = 32.71) and the power > 99% (with 99% two-sided confidence level, CL). The same effect was observed in the subgroups of girls (*P* < 10^−4^, *χ*^2^ = 16.66) and boys (*P* < 10^−3^, *χ*^2^ = 12.28). The frequency of postural defects stabilization was also significantly higher in the study group than in the control children (26.32% vs. 5.26%, *P* = 0.001, *χ*^2^ = 10.13) with power = 70% (99% CL). Conversely, postural defect progression was significantly more frequent in the control group than in young karate competitors (90.79% vs. 26.32%, respectively, *P* < 10^−8^, *χ*^2^ = 55.45). Also, in this case, the power of the test was greater than 99% with 99% CL. The differences remained significant in subgroups of girls (*P* = 10^−8^, *χ*^2^ = 29.52) and boys (*P* < 10^−5^, *χ*^2^ = 22.45).

### 3.3. Mathiass Test Analysis

The study revealed a visible difference in postural muscle strength, as measured with the Mathiass screening test. For a proper assessment, the participants stood with their upper limbs bent at the shoulder joints to 90 degrees for at least 30 seconds. In the group of children undergoing karate training, 63.16% met the time criterion without any compensations within the body. The other children yielded results between 12 and 29 seconds (mean ± SD: 22.38 ± 5.75). In the control group, 26.23% of children reached 30 seconds, while the rest of them yielded results from 12 to 27 seconds (mean ± SD: 18.83 ± 5.40) (*P* < 10^−5^). The values obtained in both groups were not dependent on age (*P* > 0.05), but these values depended on years of karate training (*r*_*s*_ = 0.34, *P* < 0.009). The participants' sex had no effect on the obtained results in the study group (*χ*^2^ = 1.04, *P* > 0.05, df = 1) or in the control group (*χ*^2^ = 0.69, *P* > 0.05, df = 1).

### 3.4. Time Spent by Children in a Sitting Position

From Monday to Friday, the examined children spent time in a sitting position for 6 to 10 hours (mean ± SD: 7.43 ± 1.03); at school, they sat for 4 to 6 hours (mean ± SD: 4.8 ± 0.44), and at home, they sat for 1 to 5 hours (mean ± SD: 2.63 ± 0.91). The results of the control group were as follows: 6–10 hours per each of the 5 working days (mean ± SD: 7.53 ± 1.19) at school (mean ± SD: 4.84 ± 0.49) and 1–5 hours at home (mean ± SD: 2.69 ± 0.99). The children's age (for the study group *P* > 0.05 and for the control group *P* > 0.05) and sex (*χ*^2^ = 3.74, *P* > 0.05, df = 6) did not affect the results. During the weekends, the boys and girls spent on average three hours less in a sitting position than they did during school (*P* < 0.00001). There were no differences between the groups (*t* = 0.75, *P* > 0.05). A detailed distribution of hours spent sitting at school and during leisure time with respect to the class the children attend is shown in Figure 3.

### 3.5. Time Spent by Children with Electronic Devices

The examined children used electronic devices regularly every day, regardless of the children's sex. The age at which they started using a mobile device or tablet for the first time ranged between 2 and 8 years (mean ± SD: 5.31 ± 1.43 years). There was no significant difference between the groups (*t* = 1.22, *P* > 0.05). The electronic devices were used between 2 and 7 days per week (mean ± SD: 4.6 ± 0.76) regardless of the child's sex (*P* > 0.05). The children spent many hours in front of a TV, PC, tablet, and mobile device. The time of use ranged between 10 and 960 minutes per week (mean ± SD: 387.19 ± 183.09) in the karate group, in comparison to the control group (*t* = 0.51, *P* > 0.05). There were correlations between device usage time and age in both groups (*r*_*s*_ = 0.31, *P* < 0.014 and *r*_*s*_ = 0.26, *P* < 0.022 for the study group and the control group, respectively). The children from the control group spent more time (and did it more often) on the internet on online portals such as Facebook than the karate children did (*t* = 2.73, *P* < 0.007). The same results were found for the amount of time spent watching TV (*t* = 4.33, *P* < 0.00002).

## 4. Discussion

The results of the present study indicate that children who regularly participated in intense karate training experienced greater improvement in posturometric parameters than other active children, even though the subjects of both groups were homogeneous in terms of age, gender, and the number of hours spent with electronic devices. Nevertheless, regression and stabilization of posture defects were observed more often in young karate competitors than in active control children in the 11-month follow-up. Conversely, postural defects progression was more characteristic for control children, and these all differences had strong statistical significance. Our study will hopefully explain what may be the cause of these changes.

Active leisure time, including regular physical activity, is one of the main goals of physioprophylaxis. The definition of physioprophylaxis of posture defects is quite new [31] and is part of comprehensive physiotherapy. Early and primary physioprophylaxis points to physical activity as the basic means of preventing the development of defects [31, 32] next to which ergonomic behaviour and the quality of everyday activities play an important role [33]. Bajorek et al. point to swimming as a form of physical activity facilitating the strengthening of weakened muscles, including the so-called postural muscles not only through active exercises and resistance training but also through weight-bearing exercises if they are required [34]. There is not much literature on the effect of systematically practiced martial arts on postural stability [35–37]. Systematically performed intensive, controlled, and specific exercise [38, 39] can reduce the risk for body posture abnormalities. Postural stability is often a key role in developing normal motor function [40].

Although the analysis of body posture in children and adolescents practicing sports is the subject of numerous studies [37, 41–44], it focuses mainly on the injuries caused by particular sports activities. However, as indicated by our own research and that of Bettany-Saltikov et al., the influence of martial arts, including karate, on posture defects in children is described only in a few reports [37, 44]. The other Polish study indicated above was conducted on a similar age group of children and adolescents, but the study focused on a detailed assessment of the sagittal plane. No statistically significant differences were found between the groups in terms of curvature, thoracic kyphosis, and lumbar lordosis. On the other hand, the study by Silkwood-Sherer et al. showed a significant deepening of both curvatures of the spine—lordosis and kyphosis—in children practising karate for at least two years, which was not found in the study of the children practising karate [45]. In the authors' study, the thoracic kyphosis in a group of karate-trained children became weaker, but within normal limits, without significant changes in the lumbar lordosis, in contrast to the control group, where the values of both angles increased. Considering the reason for this state of affairs, one may conclude that systematic exercises based on postural control such as combat sports have a direct effect on the quality of posture, which was confirmed by a test assessing the efficiency of postural muscles, a high percentage of which was within the normal range of 30 seconds, although the strength and endurance of postural muscles are insufficient in cases of deficits associated with postural control [46]. The organs involved in vision, proprioception, and the vestibular system play a key role in the registration of any deviation in the center of gravity of the body. These organs also take part in changes in the various parts of the biokinematic system. The analyzer, which is the central nervous system, determines the type of postural responses by commanding appropriate changes in muscle tension and corrections in body sway and the body segment positions in space [47]. Suitable tension and central stabilization often prevent overload and enable a more relaxed and effective execution of motor tasks while maintaining a stable posture. Stability and central stabilization training is one of the main elements in modern physiotherapy and sports.

Sports activities associated with martial arts are perfectly aligned with the designated trends in shaping and improving sensorimotor organization and central stabilization [48]. In addition, it is also important to point out movement habits based on constant exemplification of patterns repeated during a single workout and the role of sport becomes fundamental [49]. It was therefore considered whether training alone based on specific exercises can slow down postural abnormalities. This may be evidenced by the values of posturometric parameters in the frontal and sagittal planes, which despite increasing or decreasing are still within normal range.

In postural disorders, the rotational component of the body plays a very important role [47] in children practicing karate; a decrease in trunk rotation was observed. The authors were surprised by the fact that SATR scores were not dependent on training frequency and duration in both groups of subjects. And the index depended on training years only in the control group. This may indicate the fact of the quality of the exercises performed their correctness and concentration on details while performing them. Learning particular techniques used in a martial arts discipline requires the gradual mastering of successive skills after achieving previous ones as a principle of well-planned training [48]. According to the indications and algorithm of management after obtaining the SATR score [50], children with suspected scoliosis were referred to orthopedic specialists, recommending further treatment and rehabilitation. The effectiveness of karate in maintaining the correct posture was confirmed by the fact that there were no statistically significant differences in this regard and only 5 patients whose SATR increased above 7° during the one-year observation were referred to specialists, as compared to the control group in which a significant deterioration of the rotational component was observed.

When children and young people spend increasingly more time in a sitting position, active relaxation associated with physical activity is compromised. Electronics, including portable tablets and smartphones, can be used basically in all conditions and at any time. Thus, people position their body in ergonomic positions less frequently. In turn, postural asymmetries develop [31, 32].

Based on the results published in 2019 and 2020 by the WHO [2, 51], 44.4% of children spend 4 hours watching TV, and only 35.5% of children are active according to the WHO recommendations. A growing number of young people are struggling with progressive posture disorders, which may restrict the capacity of the body and consequently inhibit proper development and efficiency, demonstrating the need to develop and implement preventive and corrective activities [24, 31, 32]. This study revealed that children undergoing karate training definitely use such technology less frequently to spend time with colleagues and friends. A total of 23.88% of the children in the control group vs. 14.05% of the children undergoing karate training never met with their colleagues/friends on Facebook. Training sessions offer the possibility of direct contact during practice and beyond. Profile sport camps are frequently attended in the summer or winter holidays.

The natural need for physical activity at a young age should therefore be used to promote sports in which central stabilization is particularly emphasized. The ability to control and regulate body stability has a fundamental role in the efficient and safe execution of many activities of daily living and special motor tasks [40, 41]. As shown by our own research, group physical activity is important, especially according to the Hump Sum indicator [51].

The main factor limiting findings of the current work is the size of the study groups (*n* = 57 and *n* = 76, respectively), selected from a cohort of 1,596 children. Increasing the size of the study groups would require a much larger cohort of children, which was not feasible in our single-center study. However, we would like to emphasize that even this number of subjects was sufficient to determine the effect of karate training on posturometric parameters, both in quantitative and qualitative tests, as evidenced by very high power of the tests. The second important factor that could increase the precision of the obtained results seems to be the extension of the follow-up period to several years. In the current study, it was 11 months, although the development period of *H. sapiens* lasts much longer. For the above reasons, further research is needed, carried out on larger groups with a longer observation period. Examination of degree of sexual development characteristics would be a valuable addition to ongoing research, given the dynamic development of postural disorders during adolescence, which perhaps represents a limitation of this study, although this study by design only included children in prepubertal period. The lack of calculation of METs could also be a limitation, even though the focus of the research presented here is on posturometric parameters. Only their results can bring us closer to the answer to the question whether regular karate training influences the long-term improvement of postureometric parameters and is an effective tool preventing the manifestation of postural defects in children and adolescents.

## 5. Conclusion

Physical activity performed regularly and under the direction of a professional trainer (Sensei) can prevent postural abnormalities. In the era of a sedentary lifestyle, the number of young people with progressive postural dysfunctions, which inhibit normal psychomotor development, is increasing, demonstrating the need to develop and implement activities aimed at raising the awareness of children and their families about the effects of hypokinesis and aimed at emphasizing the advantages of systematic training. Moreover, the revealed results confirm the essential role of systematic training in posture dysfunction prevention.

## Figures and Tables

**Figure 1:** Flow diagram for selection and inclusion criteria.

**Figure 2:** The body posture assessment with classical certified tools in both groups: (a) torso rotation angle (ATR) by pediscoliometer; (b) the depth of thoracic kyphosis and lumbar lordosis angles by a digital Sunders inclinometer TMX–127; (c) the plumb line; (d) position of the scapulas; (e) Mathiass test [30].

**Figure 3:** Number distribution of hours sitting at school (top) and at home (bottom), in both groups: study (a) and control (b).

**Table 1:** Comparison of pre- and postobservation values of measured parameters in the study group (karate training children).

Parameter	First (initial) observation		Second (final) observation		*P*
	Mean ± SD (range)	95% CI	Mean ± SD (range)	95% CI	
Plumb–line anal cleft (cm)	0.24 ± 0.2 (0–0.5)	0.13–0.26	0.29 ± 0.39 (0–1.5)	0.19–0.40	>0.05^1^
Scapulae level (°)	0.98 ± 0.76 (0–2)	0.77–1.18	2.17 ± 0.96 (0–4)	1.92–2.43	<0.00001^2^
Kyphosis angle (°)	33.24 ± 3.33 (25–36)	32.36–34.13	29.31 ± 2.53 (25–35)	28.64–29.99	<0.00001^1^
Lordosis angle (°)	25.64 ± 2.08 (24–32)	25.09–26.21	25.84 ± 1.52 (22–35)	25.44–26.26	>0.05^1^
Angle of trunk rotation C_7_–Th_1_ (°)	1.47 ± 0.94 (0–3)	1.23–1.17	0.59 ± 0.82 (0–3)	0.37–0.81	<0.00001^1^
Angle of trunk rotation Th (°)	1.66 ± 1.07 (0–3)	1.38–1.95	0.82 ± 0.8 (1–3)	0.58–1.06	<0.00001^1^
Angle of trunk rotation Th-L/L (°)	1.98 ± 0.86 (1–3)	1.75–2.2	2.07 ± 0.86 (0–4)	1.84–2.29	>0.05^1^
Sum of trunk rotation SHS (°)	2.17 ± 0.82 (1–3)	1.95–2.39	2.01 ± 1.66 (0–7)	1.57–2.45	>0.05^2^

^1^Wilcoxon signed-rank test for continuous variables with nonnormal distribution; ^2^Student's *t* test for continuous variables with normal distribution; abbreviations: C: cervical spine; Th: thoracic spine; L: lumbar spine, Th–L: thoraco–lumbar spine; NORM of: plumb line anal cleft (0-0.5 cm), scapulae level (0-2°), kyphosis and lordosis angle (24-36°), angle of trunk rotation C_7_ – Th_1_ (0-3°), angle of trunk rotation Th (0-3°), and angle of trunk rotation Th-L/L (0-3°).

**Table 2:** Comparison of pre- and postobservation values of measured parameters in the control group (active children).

Parameter	First (initial) observation		Second (final) observation		*P*
	Mean ± SD (range)	95% CI	Mean ± SD (range)	95% CI	
Plumb–line anal cleft (cm)	0.37 ± 0.21 (0–0.5)	0.32–0.42	0.71 ± 0.53 (0–2)	0.59–0.83	<0.00001^1^
Scapulae level (°)	0.69 ± 0.68 (0–2)	0.54–0.85	0.38 ± 0.84 (0–4)	0.19–0.57	<0.001^1^
Kyphosis angle (°)	30.02 ± 3.1 (24–36)	29.31–30.73	32.29 ± 4.5 (23–42)	31.26–33.32	<0.00001^2^
Lordosis angle (°)	31.42 ± 2.46 (24–32)	30.86–31.98	32.87 ± 1.89 (22–35)	32.44–33.31	<0.00001^2^
Angle of trunk rotation C_7_–Th_1_ (°)	1.84 ± 0.89 (1–3)	1.63–2.04	2.84 ± 1.33 (0–6)	2.59–3.19	<0.00001^2^
Angle of trunk rotation Th (°)	2.54 ± 0.7 (1–3)	2.38–2.69	3.59 ± 1.85 (0–7)	3.17–4.02	<0.00001^2^
Angle of trunk rotation Th-L/L(°)	2.35 ± 0.81 (1–3)	2.17–2.54	3.19 ± 1.93 (1–7)	2.76–3.64	<0.00001^2^
Sum of trunk rotation SHS (°)	2.77 ± 0.41 (2–3)	2.68–2.87	5.68 ± 1.81 (0–9)	5.27–6.09	<0.00001^2^

^1^Wilcoxon signed-rank test for continuous variables with nonnormal distribution; ^2^Student's *t* test for continuous variables with normal distribution; abbreviations: C: cervical spine; Th: thoracic spine; L: lumbar spine, Th–L: thoraco–lumbar spine; NORM of: plumb line anal cleft (0-0.5 cm), scapulae level (0-2°), kyphosis and lordosis angle (24-36°), angle of trunk rotation C_7_–Th_1_ (0-3°), angle of trunk rotation Th (0-3°), and angle of trunk rotation Th-L/L (0-3°).

**Table 3:** Percentage values of body postural defects regression, stabilization, and progression in the study group (karate training children) and the control group (active children).

Group	Sex	*n*	Postural defects					
			Regression		Stabilization		Progression	
			*n*	%	*n*	%	*n*	%
Study group	Girls	33	17^∗^	51.52	8^∗∗^	24.24	8^∗^	24.24
	Boys	24	10^∗^	41.67	7^∗∗^	29.17	7^∗^	29.17
	Both sexes	57	27^∗^	47.36	15^∗^	26.32	15^∗^	26.32
Control group	Girls	32	1	3.13	1	3.13	30	93.75
	Boys	44	2	4.58	3	6.82	39	88.64
	Both sexes	76	3	4.11	4	5.26	69	90.79

^∗^ *P* < 0.05 vs. control group. ^∗∗^Not statistically significant (*P* > 0.025) after Bonferroni correction vs. control group.

## Data Availability

The raw data used to support the findings of the present research are available from the corresponding author upon request.
